# Deep Learning-Based Digital Subtraction Angiography Characteristics in Nursing of Maintenance Hemodialysis Patients

**DOI:** 10.1155/2022/9356108

**Published:** 2022-08-27

**Authors:** Jinyan Mi

**Affiliations:** Blood Dialysis Room, Tonglu Hospital of Traditional Chinese Medicine, Tonglu, Hangzhou 311500, Zhejiang, China

## Abstract

This study is aimed at exploring the diagnostic value of digital subtraction angiography (DSA) based on faster region-based convolutional networks (Faster-RCNN) deep learning for maintenance hemodialysis (MHD) diseases and to provide a theoretical basis for clinical nursing. A total of 50 MHD patients who were clinically diagnosed in the Blood Purification Center were randomly divided into the control group and the experimental group (25 cases for each group). The control group was given routine nursing intervention, and the experimental group was given overall nursing intervention under the supervision of DSA. A faster RCNN multitarget detection network was constructed to analyze the average accuracy of various vascular structures in the test set. The self-rating anxiety scale (SAS) and self-rating depression scale (SDS) were used to evaluate the degree of anxiety and depression. The urine volume before and after the operation, local hematoma after a puncture, the incidence of complications, and nursing satisfaction were recorded. The results showed that the average accuracy of the vein, internal carotid artery, circle of Willis, venous sinus, and venous vessels was 0.876, 0.916, 0.994, 0.925, and 0.732, respectively. The success rate of surgery in the experiment group was higher than that in the control group, and the difference had statistical significance (*P* < 0.05). The SAS score and SDS score in the experimental group were significantly lower than those in the control group (*P* < 0.05). The total incidence rate of complications in the experimental group (16.00%) was significantly lower than that in the control group (44.00%) (*P* < 0.05). The satisfaction rate of the experimental group was significantly higher than that of the control group (*P* < 0.05). The Faster-RCNN model had the best effect in differentiating the circle of Willis and a poor effect in differentiating venous vessels. DSA based on Faster-RCNN can significantly improve the success rate of puncture in MHD patients. The implementation of holistic nursing intervention under its supervision can significantly reduce postoperative complications and improve patient satisfaction with nursing compared with routine nursing.

## 1. Introduction

An arteriovenous fistula (AVF) is a procedure before maintenance hemodialysis (MHD) in which an artery is surgically connected to a vein so that the vein better processes the amount of blood returned to the body [1–3]. Many complications occur in patients undergoing MHD; for example, factors such as arteriosclerosis, repeated puncture, and infection can cause intimal hyperplasia or embolism, which leads to stenosis or occlusion of AVF vessels in patients, seriously affecting the patency of vessels and reducing fistula blood flow [4–6].

When it is suspected that the blood flow of AVF is reduced in MHD patients, examination and diagnosis and treatment must be performed as early as possible, and digital subtraction angiography (DSA) is an important means to understanding the vascular function of AVF [7]. DSA is a digital subtraction technique based on sequential images, which obtains the difference part by subtracting two frames of images in the same part of the human body, eliminates bone and soft tissue structures, makes the vessels filled with contrast agent in the second frame appear in the subtraction map, and enhances the contrast [8–10]. DSA is of great significance in the clinical diagnosis of vascular diseases. It is the most effective detection method in the interventional diagnosis and treatment of cardiovascular and cerebrovascular diseases and is the “gold standard” for the diagnosis of vascular diseases [11, 12]. In recent years, deep learning has been widely used in the field of image processing by virtue of its ultra-high prediction accuracy in recognition applications, and the use of deep learning to process some tasks is simpler and more effective than other algorithms. Faster-RCNN is optimized based on RCNN and Fast-RCNN. Structurally, Faster-RCNN integrates feature extraction, proposal extraction, bounding box regression, and classification into the same network, which greatly improves the comprehensive performance and is especially obvious in terms of detection speed. The automatic discrimination of DSA based on deep learning mainly includes structural and temporal information. For the analysis of structural information of DSA, artificial labeling of vascular structures is often used, and then the performance characteristics of the labeling site are extracted to continue the next exploration and analysis [13–15]. At present, there are few studies related to the temporal information discrimination of DSA sequences, which has the potential value for clinical research and application.

Most MHD patients have serious physiological and psychological dysfunction. While suffering from the disease, patients are burdened with heavy economic pressure, so they are prone to developing many psychological problems including anxiety, depression, etc. These negative emotions greatly affect the progress and quality of hemodialysis work, resulting in increased difficulty in nursing work. Holistic nursing is an emerging nursing work mode, which is guided by modern nursing concepts, centered on nursing procedures, and systematizes all aspects of clinical nursing and nursing management. In addition to strengthening the attention to patients, nursing staff also need to focus on the environment, psychological state, physical factors, and other factors affecting the rehabilitation of the disease. The goal is to provide the best care suitable for people according to their physical, psychological, social, cultural, spiritual, and other needs in order to achieve the purpose of treating the disease.

Under the visual image of DSA based on a deep learning algorithm, 50 MHD patients who were clinically diagnosed with weakened or disappeared fistula vascular tremor in the Blood Purification Center from May 2019 to October 2021 were randomly divided into the control group and the experimental group. The purpose was to explore the automatic identification and localization of key vascular structures by DSA sequence examination and to provide technical support for the automation of DSA interpretation. In addition, it was to explore its diagnostic value for autologous AVF in MHD patients and to provide a theoretical basis for clinical nursing.

## 2. Materials and Methods

### 2.1. Study Subjects

Fifty MHD patients who were clinically confirmed to have weakened or disappeared tremors of fistula vessels in the hospital from May 2019 to October 2021 were selected, and the blood flow of the patients with autologous AVF decreased (blood flow <150 mL/min). They were randomly divided into the control group (25 cases, routine nursing) and the experimental group (25 cases, overall nursing intervention); 28 males and 22 females, with an average age of (53.4 ± 12.5) years. The service life of AVF was 1–4 years. There was no significant difference in basic information between the two groups (*P* > 0.05). The experiment was approved by the ethics committee of the hospital, and the patients and their families understood the situation and signed the informed consent.

Inclusion criteria: patients receiving MHD treatment for more than 1 month; MHD and establishment of AVF were performed; patients with normal cognitive function and clear language expression.

Exclusion criteria: patients under 18 years of age; patients with infectious diseases; patients with mental diseases; patients allergic to contrast medium.

### 2.2. Test Method

Preparation before the examination: the patients patiently introduced the precautions in the examination, the patients' tension was paid attention to at any time, and the patients were informed not to move the examined limb at will during the examination to avoid damaging the blood vessels and affecting the imaging results. The routine withdrawal of 1 mL of stock solution for skin tests was required before the examination to avoid severe allergic reactions due to the contrast medium.

Angiographic examination: percutaneous radial artery angiography was performed in all hemodialysis patients using a mobile flat-detector C-arm machine. 18G internal fistula puncture needle was used. Before puncture, 5% povidone-iodine was used to disinfect 8-10 cm around the punctured skin. About 2 cm of the internal fistula was punctured. After the completion, 15–30 mL nonionic contrast agent ioversol was injected using a high-pressure syringe.

Post treatment after angiography: after the completion of angiography, the puncture nurse performed compression bandaging on the local wound, and high-flux hemodialysis was performed for 4 hours on the day after the examination.

### 2.3. Nursing Methods

Patients in the control group received routine nursing intervention, the examination was carefully completed, patients were given appropriate care; patients were helped change dressing according to the doctor's requirements; and once an abnormal situation was found, the doctor was immediately reported.

In the experimental group, patients were given overall nursing intervention under the supervision of DSA, and appropriate nursing measures were given at admission, during operation, post operation, and at discharge. At admission, patients were introduced to the basic information of attending physicians and nurses, patients' clinical information was understood in detail, and patients' questions were actively answered. During the operation, the patient's vital signs were paid attention to and the patients were encouraged. After surgery, the patient's incision bleeding, exudation, and pain were paid attention to, and the doctor was reported at any time. At discharge, the patients were advised to take proper physical activity and return to the clinic at 3 to 6 months.

### 2.4. Outcome Measures

The self-rating anxiety scale (SAS) and self-rating depression scale (SDS) were used to evaluate the degree of anxiety and depression, respectively [16]. Both scales contain 20 items, both of which are 4-grade scoring, with 10 points for each item. The higher the score, the more serious the anxiety and depression. Preoperative and postoperative urine volume, local hematoma after a puncture, the incidence rate of complications, and nursing satisfaction were observed and recorded.

### 2.5. DSA Image Analysis

In the test set of 50 MHD patients, the overexposed images were excluded, and 2–3 frames of images were selected from each case. 126 internal carotid arteries, 234 circles of Willis, 150 large veins, 145 venous vessels, and 162 venous sinuses were labeled. From a total of 180, 96 served as the test set and 84 served as the training set. The main vessel location information of the anteroposterior image of the internal carotid artery was labeled by a professional physician. The pictures of the late arterial phase and venous sinus phase were mainly labeled, in which the internal carotid artery and circle of Willis were mainly labeled in the arterial phase image (Figure 1(a)); the large veins and venous drainage vessels were labeled in the venous sinus phase image (Figure 1(b)). The labeled vessel category and coordinate position were saved to the corresponding XML file, and all the data were made into a dataset (VOC2007 format) for training.

### 2.6. Faster Region-Based Convolutional Networks (Faster-RCNN) Algorithm

The faster-RCNN algorithm was composed of a basic feature extraction module, a region prediction network module, and a classification regression module [17].  Figure 2 shows the basic flow of faster-RCNN processing images. The samples of DSA sequences were labeled to construct a multitarget detection Faster-RCNN network, using Resnet50 as the infrastructure. Picture features were extracted to train the detection model, and the optimal model was selected to detect various types of vessels. The faster-RCNN-based flow of the DSA detection algorithm is shown in Figure 3.

### 2.7. Evaluation Index of Simulation Experiment

The average value and average precision (AP) were used to evaluate the algorithm detection results. AP is an evaluation index to measure the classification results in multilabel classification, which refers to the area under the precision-recall (P-R) curve. In general, for the data set of *n* samples, the real label and prediction probability of each sample were calculated, and finally, the average was performed. A larger AP value indicated better classifier performance.

### 2.8. Statistical Methods

All experimental data were statistically analyzed by the SPSS 20.0 software. Measurement data were expressed as the mean + standard deviation ($\bar{\text{x}}$ ± *s*). Enumeration data were statistically inferred by the *χ*^2^ test. Measurement data conformed to a normal distribution and a *t*-test was used. *P* < 0.05 was considered statistically significant.

## 3. Results

### 3.1. Faster-RCNN Model Establishment Analysis

The AP of the labeled internal carotid artery, circle of Willis, large vein, venous vessel, and venous sinus was statistically analyzed using the trained Faster-RCNN model (Figure 4). The results showed that the AP of the vein was 0.876, the AP of the internal carotid artery was 0.916, the AP of the circle of Willis was 0.994, the AP of the venous sinus was 0.925, and the AP of the venous vessels was 0.732. Analysis of AP values suggested that the faster-RCNN model was the best for differentiating the circle of Willis and poor for differentiating venous vessels. The faster-RCNN model had a good effect on the detection of various vascular structures.

### 3.2. Visualization Result Analysis of Structure Identification of DSA Image

According to the results of image visualization, the location of the internal carotid artery and the circle of Willis can be detected in the arterial phase in the faster-RCNN model (Figures 5(a)–5(c)). The location of large veins and venous vessels can be detected in the venous phase (Figures 5(d)–5(f)).

### 3.3. Success Rate of Puncture

Fifty MHD patients successfully completed the contrast examination, 39 patients were successful in one puncture, and 6 patients were successful in the second puncture after adjusting the direction and depth of the puncture needle. The success rate of primary puncture and secondary puncture in the experimental group was significantly higher than that in the control group, and the differences had statistical significance (*P* < 0.05). The difference in the success rate of operations between the two groups had statistical significance (*P* < 0.05) (Table 1).

### 3.4. Comparison of Depression and Anxiety

The SAS score of the experimental group was (28.67 ± 5.72) points, while that of the control group was (37.68 ± 6.28) points. The experimental group was significantly lower than the control group, and the difference had statistical significance (*P* < 0.05). The SDS score of the experimental group (32.36 ± 8.76) was significantly lower than (45.62 ± 9.78) of the control group, and the difference had statistical significance (*P* < 0.05) (Figure 6).

### 3.5. Changes in Urine Volume before and after Angiography

Before and after angiography, there was no significant difference in urine volume between the two groups (*P* > 0.05) (Table 2).

### 3.6. Comparison of Complications

The total incidence of complications in the experimental group (16.00%) was significantly lower than (44.00%) in the control group, and the difference was statistically significant (*P* < 0.05). In the control group, 2 cases of pseudoaneurysm, 3 cases of perivascular hematoma, 1 case of subcutaneous emphysema, and 5 cases of nerve injury were found; 1 case of pseudoaneurysm, 2 cases of perivascular hematoma, and 1 case of nerve injury were found in the experimental group (Table 3).

### 3.7. Comparison of Nursing Satisfaction Rate

In the experimental group, there were 24 cases of satisfaction and 1 case of dissatisfaction, and the nursing satisfaction was 96.00%. In the control group, there were 21 cases of satisfaction and 3 cases of dissatisfaction, and the nursing satisfaction was 84.00%. The satisfaction of patients in the experimental group was significantly higher than that of patients in the control group, and the difference was statistically significant (*P* < 0.05).

## 4. Discussion

MHD access is the lifeline of treatment for patients with end-stage renal disease, but it is easy to have narrow and blocked vascular access during treatment, resulting in significantly reduced hemodialysis flow, seriously affecting the final therapeutic effect and prognosis of patients [18–20]. Balloon dilatation of AVFs, as the treatment of choice for MHD, is widely used in clinical practice because of its characteristics of less susceptibility to infection and a long duration of patency [21–23].

The imaging of DSA is intuitively clear; less contrast medium is used, a small amount of X-ray radiation and even small vessels can be clearly displayed. However, the disadvantage of DSA is that the field of view is small [24, 25]. Starting from the two aspects of structural information and temporal information, the phase of cerebrovascular DSA was automatically identified for the first time. On the test set, venous AP was 0.876, internal carotid artery AP was 0.916, circle of Willis AP was 0.994, venous sinus AP was 0.925, and venous vascular AP was 0.732. Analysis of AP values suggested that the Faster-RCNN model had the best discrimination performance for the circle of Willis and poor discrimination performance for venous vessels. Yamuna et al. (2017) [26] concluded that when the hemodynamic parameters of patients with end-stage renal disease are low, active therapeutic intervention should be initiated as early as possible. DSA-guided balloon dilatation of AVF can be performed without contrast medium and without damage to the kidney, which is of great significance in improving the quality of life of MHD patients. DSA has some disadvantages, some patients are allergic to the contrast agent, severe cases will produce anaphylactic shock, and it may cause puncture site bleeding or infection. However, it can accurately show the distribution of blood vessels under computer vision images, so as to more clearly understand the extent and degree of vascular diseases, improve the accuracy of vascular disease diagnosis, and provide a safe and accurate guarantee for further interventional therapy.

The success rate of primary puncture and secondary puncture in the experimental group was significantly higher than that in the control group, and the difference had statistical significance (*P* < 0.05). The difference in the success rate of operations between the two groups had statistical significance (*P* < 0.05). The reason was that the balloon dilatation of AVF based on DSA can accurately obtain the specific situation of the fistula vessels in the body, can visually understand the blood flow of the feeding artery and reflux vein, and accurately locate the extravascular structure and vessel wall, improving the success rate of puncture [27, 28]. In the control group, 2 cases of pseudoaneurysm, 3 cases of perivascular hematoma, 1 case of subcutaneous emphysema, and 5 cases of nerve injury were found; in the experimental group, 1 case of pseudoaneurysm, 2 cases of perivascular hematoma, and 1 case of nerve injury were found. The total incidence rate of complications in the experimental group was significantly lower than that in the control group, and the difference had statistical significance (*P* < 0.05). The reason may be that the main approach for conventional balloon dilatation of AVFs is the distal end of the radial artery, while the distal site of the radial artery has more vascular branches. DSA enables flexible adjustment of the puncture site according to the needs and reduces the occurrence of complications such as nerve injury and pseudoaneurysm, which is consistent with the results of Fujimoto et al. (2020) [29].

The patients were given comprehensive nursing at each stage, and nursing intervention was performed from physical, psychological, and social aspects. The results showed that the SAS score and SDS score in the experimental group were lower than those in the control group (*P* < 0.05); the satisfaction rate in the experimental group was higher than that in the control group (*P* < 0.05). It indicated that the nursing staff combined with psychological nursing intervention during nursing work.

## 5. Conclusion

MHD patients who were clinically diagnosed in the Blood Purification Center were randomly divided into the control group and the experimental group to investigate the diagnostic value of DSA for autogenous AVF in MHD patients. The faster-RCNN model had the best differential performance for the circle of Willis and poor differential performance for venous vessels. DSA-guided balloon dilatation of venous fistulas based on Faster-RCNN significantly improved the success rate of puncture in MHD patients, reduced postoperative complications, and improved patient satisfaction. However, there are still some shortcomings; for example, the sample size is small, resulting in insufficient data, which needs to be continuously improved in future work. More comprehensive samples and more mature experimental protocols will be applied to explore this direction in depth in the future. In conclusion, it provides an experimental and theoretical basis for the clinical application of faster-RCNN-based DSA.

## Figures and Tables

**Figure 1:** Angiographic image. (a) Arterial phase labeling, the red boxes are the internal carotid artery and circle of Willis, (b) venous sinus phase labeling, the red boxes are venous sinuses, large veins, and venous draining vessels.

**Figure 2:** Flow of faster-RCNN processing image.

**Figure 3:** Flow of faster-RCNN-based DSA vessel detection algorithm.

**Figure 4:** P-R curve corresponding to the vascular characteristic region and corresponding AP value.

**Figure 5:** Detection results of vascular images at different stages. (a) Early arterial detection results, artery, and circle of Willis; (b) midterm arterial detection results, artery, and circle of Willis; (c) late arterial detection results, artery, and circle of Willis; (d) early venous detection results, large vein, and venous vessel; (e) midterm venous detection results, large vein, and venous vessel; and (f) late venous detection results, large vein, and venous vessel.

**Figure 6:** Comparison of anxiety and depression between two groups. ^*∗*^Compared with the control group, *P* < 0.05.

**Table 1:** Success rate of puncture in two groups of MHD patients (*n*, %).

Item	Control group (*n* = 25)	Experimental group (*n* = 25)	*χ* ^2^	*P*
One-time puncture success rate	19 (76.00)	20 (80.00)	5.362	<0.05
Two-time puncture success rate	2 (8.00)	4 (16.00)	2.281	<0.05
Surgical success rate	21 (84.00)	24 (96.00)	3.271	<0.05

**Table 2:** Changes in urine volume before and after angiography ($\bar{\text{x}}$ ± *s*, mL).

Angiography time	Control group (*n* = 25)			Experimental group (*n* = 25)		
	0–500 mL	500–1000 mL	>1000 mL	0–500 mL	500–1000 mL	>1000 mL
Before angiography	356.7 ± 120.1	736.2 ± 150.2	1241.5 ± 241.5	348.7 ± 132.4	743.4 ± 163.2	1321.5 ± 243.5
After angiography	342.6 ± 138.4	721.2 ± 153.2	1128.8 ± 237.6	341.8 ± 136.2	732.1 ± 152.3	1235.3 ± 256.1
*P*	>0.05	>0.05	>0.05	>0.05	>0.05	>0.05

**Table 3:** Comparison of complications (*n*, %).

Item	Control group (*n* = 25)	Experimental group (*n* = 25)	t/*χ*^2^	*P*
Pseudoaneurysm	2 (8.00)	1 (4.00)	2.576	0.0347
Perivascular hematoma	3 (12.00)	2 (8.00)	2.738	0.0462
Subcutaneous emphysema	1 (4.00)	0 (0.00)	2.462	0.0416
Nerve injury	5 (20.00)	1 (4.00)	2.048	0.0286
Total incidence	11 (44.00)	4 (16.00)	2.498	0.0127

## Data Availability

The data used to support the findings of this study are available from the corresponding author upon request.
